The article "Long noncoding RNA MALAT1 promotes the stemness of esophageal squamous cell carcinoma by enhancing YAP transcriptional activity" was retracted in 2023. Reasons: duplicated images; signs of a paper mill; unreliable results or conclusions.

# Long noncoding RNA MALAT1 promotes the stemness of esophageal squamous cell carcinoma by enhancing YAP transcriptional activity

**DOI:** 10.1002/2211-5463.12676

**Published:** 2019-06-11

**Authors:** Qi Yao, Jun Yang, Ting Liu, Jianjiang Zhang, Yibo Zheng

**Affiliations:** ^1^ Department of Geriatric Medicine Ningbo First Hospital China

**Keywords:** esophageal squamous cell carcinoma, MALAT1, migration, stemness, YAP

## Abstract

The tumor promoting roles of long noncoding RNA (lncRNA) MALAT1 have been revealed in various cancers; however, its roles in esophageal squamous cell carcinoma (ESCC) have not previously been disclosed. In this study, we found that MALAT1 expression was remarkably increased in ESCC cells compared to normal human esophageal epithelial cells. In addition, knockdown of MALAT1 attenuated the stemness of ESCC cells, as evidenced by a decrease in spheroid formation capacity, stemness marker expression and aldehyde dehydrogenase 1 activity. Moreover, MALAT1 knockdown decreased the migration ability of ESCC cells. Notably, knockdown of MALAT1 enhanced the radiosensitivity and chemosensitivity of ESCC cells. We also established that MALAT1 binds directly to Yes‐associated protein (YAP), thereby enhancing YAP protein expression and increasing YAP transcriptional activity. Overexpression of YAP partially rescued the effect of MALAT1 knockdown on stemness and radiosensitivity of ESCC cells. Overall, this study has identified that a novel MALAT1–YAP axis promotes the stemness of ESCC cells, and thus could be a potential target for treatment of ESCC.

**Abbreviations**
ALDH1: aldehyde dehydrogenase 1
CSC: cancer stem cell
ESCC: esophageal squamous cell carcinoma
HEEC: human esophageal epithelial cell
LncRNA: long noncoding RNA
qRT‐PCR: quantitative real‐time PCR
RIP: RNA immunoprecipitation
SD: standard deviation
TNBC: triple negative breast cancer
YAP: Yes‐associated protein

Esophageal cancer is classified into squamous cell carcinoma and adenocarcinoma, among which esophageal squamous cell carcinoma (ESCC) accounts for more than 90% of cases in China 1. Most of the patients with ESCC are identified only in the middle and advanced stages, missing the right time for surgery, and radiotherapy and chemotherapy alone cannot significantly improve the quality of life for ESCC patients 2. Therefore, it is essential to find novel targets which could facilitate the development of the treatment of ESCC.

Cancer stem cells (CSCs), also called tumor initiating cells, are regarded as the origin of cancer development and progression. A lot of work has attempted to identify potential CSC‐targeting drugs. For example, recent work has disclosed that dasatinib enhances the chemotherapeutic sensitivity of triple negative breast cancer (TNBC) cells by targeting breast CSCs and could be used in combination with paclitaxel to overcome chemoresistance in TNBC 3. Venetoclax disrupts the energy metabolism of leukemia stem cells with azacitidine in patients with acute myeloid leukemia 4. Smoothened inhibitors could target breast CSCs and thus sensitize TNBC cells to docetaxel, improving survival and reducing metastatic burden in the phase I clinical trial EDALINE 5. However, there are no drugs that are used to effectively kill CSCs in the clinic, indicating the importance of revealing other factors contributing to the stemness of tumors.

The article "Long noncoding RNA MALAT1 promotes the stemness of esophageal squamous cell carcinoma by enhancing YAP transcriptional activity" was retracted in 2023. Reasons: duplicated images; signs of a paper mill; unreliable results or conclusions.

Increasing evidence shows that long noncoding RNAs (lncRNAs) play important roles in regulating the stemness of cancer cells. For example, lncRNA CASC11 promotes the stemness of small cell lung cancer cells and predicts postoperative survival probably by promoting transforming growth factor β1 expression 6. LncRNA BCAR4 maintains the stemness of colorectal cancer cells by sponging miR‐655 and thus activating STAT3 signaling 7. Mesenchymal stem cells could induce lncRNA MACC1‐AS1 expression, which promotes the fatty acid oxidation‐dependent stemness of gastric cancer cells 8. LncRNA MALAT1 has been revealed to promoter cancer progression in different cancers. For example, MALAT1 promotes the progression of glioma cells by suppressing the miR‐129–TGIF2 axis 9. MALAT1 potentiated the epithelial–mesenchymal transition and angiogenesis by regulating miR‐126‐5p activity in colorectal cancer 10. However, MALAT1 has been shown to suppress breast cancer metastasis in a MALAT1‐knockout mice model 11. These results suggest that MALAT1 may have opposite effects in different tumors. Notably, previous studies have shown that MALAT1 might be a predictive marker of poor prognosis in patients who underwent radical resection of middle thoracic ESCC 12. Additionally, MALAT1 promotes the migration and proliferation in ESCC 13, 14. However, its effects on the progression of ESCC remain unclear.

Yes‐associated protein (YAP), as the critical effector of the Hippo pathway, could promote the progression of CSCs 15, 16. In addition to being regulated by the upstream Hippo pathway, YAP activity is regulated by other factors, for example, statin blocks the YAP–CD44 axis and subsequently attenuates the stemness of malignant mesothelioma cells 17. AKAP–Lbc/Rho signaling sustains the nuclear function of YAP by modulating the organization of actin microfilaments 18. Additionally, recent studies have revealed that lncRNAs could modulate YAP activity by regulating the upstream effectors of YAP 19, 20. Notably, lncRNA MALAT1 could regulate the activity of transcriptional factors 21, 22, 23, 24. In this investigation, we have found that lncRNA MALAT1 could directly bind to YAP, thereby enhancing YAP transcriptional activity and promoting the stemness of ESCC cells.

The article "Long noncoding RNA MALAT1 promotes the stemness of esophageal squamous cell carcinoma by enhancing YAP transcriptional activity" was retracted in 2023. Reasons: duplicated images; signs of a paper mill; unreliable results or conclusions.

## Materials and methods

### Cell culture and reagents

ESCC cell lines Eca‐109 and TE‐1, as well as normal human esophageal epithelial cells (HEEC) were purchased from the Cell Bank of Chinese Academy of Sciences (Shanghai, China). The cells were cultured in 1640 medium (Thermo Fisher Scientific, Waltham, MA, USA) containing 10% FBS (Thermo Fisher Scientific), 80 U·mL^−1^ penicillin and 0.08 mg·mL^−1^ streptomycin under a humidified atmosphere with 5% CO_2_ at 37 °C.

### Lentivirus package

A lentivirus package was constructed by OBiO Inc. (Shanghai, China). The knockdown lentivirus vector for MALAT1 and overexpression vector for YAP were designated as Len‐MALAT1‐KD and Len‐YAP‐OE, respectively. Also, empty lentivirus vector was utilized as a control group.

### Quantitative real‐time PCR

Total RNA was extracted from cells using TRIzol reagent (Thermo Fisher Scientific) following the manufacturer's recommendations. Then, cDNA was reverse synthesized using HiScript® Q Select RT SuperMix for qPCR (Vazyme, Nanjing, China) according to the standard procedure. mRNA expression levels were measured with AceQ® Universal SYBR® qPCR Master Mix (Vazyme) on LightCycler® 480 (Roche, Basel, Switzerland). Glyceraldehyde 3‐phosphate dehydrogenase was used as an internal reference. The relative expression levels of mRNA were calculated using the $2{}^{-\Delta \Delta C_{t}}$ method.

### Western blot

Cells were lysed, and the total protein was extracted using a whole protein extraction kit (cat. no. KGP2100; KeyGEN BioTECH, Nanjing, China). The protein concentration was measured using a BCA Protein Assay Kit (cat. no. KGP902, KeyGEN BioTECH). Twenty micrograms of protein was separated by SDS/PAGE and transferred onto poly(vinylidene difluoride) membranes (Merck Millipore, Billerica, MA, USA), which were followed by incubating with 10% non‐fat milk at room temperature for 1.5 h. Then the membranes were incubated with the corresponding primary antibodies overnight at 4 °C followed by incubating with secondary horseradish peroxidase‐labeled goat anti‐rabbit IgG(H + L) or horseradish peroxidase‐labeled goat anti‐mouse IgG(H + L) (Beyotime, Beijing, China) for 1 h at room temperature. An ultra‐sensitive ECL chemiluminescence kit (Beyotime) was used to detect the signal on a Tanon 5200 machine (Tanon, Shanghai, China).

### Analysis of the formation of spheroid

ESCC cells were cultured in ultra‐low attachment 24‐well plates (Corning, Union City, CA, USA) at 1000 cells/well with Dulbecco's modified Eagle's medium/F12 medium supplemented with 1 × B27 (Sigma‐Aldrich, St Louis, MO, USA), 20 ng·mL^−1^ bFGF (MedChemExpress, Monmouth Junction, NJ, USA), 20 ng·mL^−1^ epidermal growth factor (MedChemExpress) and antibiotics at 37 °C under a 5% humidified CO_2_ atmosphere. After 10 days, the number and size of spheroids were evaluated and quantified under a microscope.

The article "Long noncoding RNA MALAT1 promotes the stemness of esophageal squamous cell carcinoma by enhancing YAP transcriptional activity" was retracted in 2023. Reasons: duplicated images; signs of a paper mill; unreliable results or conclusions.

### Transwell migration assay

The detailed procedure of the Transwell migration assay is discussed in a previous study 25. Briefly, ESCC cells following different treatments were digested and re‐suspended, and 8 × 10^4^ cells were added to each of the upper chambers of a 24‐well plate containing MILLIcell PET Hanging Cell Culture Inserts with a pore size of 8 μm PET (Millipore). Eight hundred microliters of medium containing 20% FBS was used as a chemo‐attractant in the bottom chamber. After 24 h, the cells migrating into the bottom chamber were fixed in methanol for 15 min and stained with 0.1% crystal violet for 15 min. Five random fields from each well were counted in triplicate by using a phase contrast microscopy. Quantification was carried out with a microplate reader (*D*_570nm_) after destaining with 30% glacial acetic acid.

### RNA immunoprecipitation

RNA immunoprecipitation (RIP) analysis was performed using EZ‐Magna RIP™ RNA‐Binding Protein Immunoprecipitation Kit (Merck Millipore) following the manufacturer's recommendation.

### Luciferase reporter assay

A luciferase reporter assay was performed to detect the activity of YAP promoter and 8xGTIIC‐luciferase plasmid (Plasmid no. 34615), a YAP‐responsive synthetic promoter driving luciferase expression plasmid purchased from Addgene (Watertown, MA, USA). The promoter sequences of YAP were inserted into the pGL3‐promoter vector, which was designated as pGL3‐YAP. Then, 8xGTIIC‐luciferase plasmid or pGL3‐YAP was co‐transfected with β‐gal into ESCC cells following the infection of Len‐MALAT1‐KD. After 72 h, the cells were collected, and luciferase activity was determined by ONE‐Glo™ + Tox Luciferase Reporter and Cell Viability Assay kit (E7110) (Promega, Madison, WI, USA) and VivoGlo Luciferin‐β‐gal Substrate kit (P1061) (Promega). The β‐gal activity was used for normalization.

### ALDH1 activity assay

Aldehyde dehydrogenase 1 (ALDH1) activity was detected using ALDH Activity Assay Kit (Colorimetric) (cat. no. KA3742; Abnova, Taipei, Taiwan, China) following the manufacturer's protocols.

### Cell viability analysis

For a chemosensitivity assay, ESCC cells were cultured in 96‐well plates at 3000 cells/well following by subjecting them to cisplatin (cat. no. HY‐17394; MedChemExpress) treatment for 24, 48, and 72 h. For radiosensitivity, the cells were treated with 3.2 Gy·min^−1^ by 6MV‐X‐ray Vertical Direct radiation using a Varian 2300EX Linear Accelerator, where the source skin distance is 100 cm for 24, 48, and 72 h. The cell viability was examined by using an Enhanced Cell Counting Kit‐8 (cat. no. C0041; Beyotime) according to the manufacturer's protocols.

The article "Long noncoding RNA MALAT1 promotes the stemness of esophageal squamous cell carcinoma by enhancing YAP transcriptional activity" was retracted in 2023. Reasons: duplicated images; signs of a paper mill; unreliable results or conclusions.

### Statistical analysis

All the obtained data are represented as mean ± standard deviation (SD). Analysis of the datasets with only two groups was performed using Student's *t*‐test. The differences between the groups were analyzed using one‐way ANOVA with the Tukey–Kramer *post hoc* test, and *P* < 0.05 was considered to be significant.

## Results

### Knockdown of MALAT1 attenuates the stemness of ESCC cells

The expression of MALAT1 in ESCC cells and HECCs was first detected and it was found that MALAT1 expression was remarkably increased in ESCC cells compared to HECCs (Fig. 1A). As CSCs contribute to tumor progression, there is a possibility that MALAT1 could be engaged in the stemness of ESCC cells. MALAT1 was knocked down in ESCC cells owing to its higher expression level in ESCC cells. The knockdown efficiency of Len‐MALAT1‐KD was confirmed by a quantitative real‐time PCR (qRT‐PCR) assay in ESCC cells (Fig. 1B). As expected, knockdown of MALAT1 reduced the expression of stemness markers (SOX2 and Nanog) in ESCC cells (Fig. 1C–E). Additionally, the capacity of spheroid formation was attenuated by knockdown of MALAT1 in ESCC cells, which was evident from the decrease in the size (Fig. 1F) and number (Fig. 1G) of the spheroids. Moreover, ALDH1 activity was reduced by MALAT1 as well (Fig. 1H).

**Figure 1:** Knockdown of MALAT1 attenuates the stemness of ESCC cells. (A) MALAT1 level was examined in ESCC cells and HEECs by qRT‐PCR assay. (B) The knockdown efficiency of len‐MALAT1‐KD was confirmed in ESCC cells by qRT‐PCR analysis. (C, D) The mRNA levels of stemness markers (SOX2 and Nanog) were detected in ESCC cells with or without MALAT1 knockdown. (E) The protein level of stemness markers (SOX2 and Nanog) was determined in ESCC cells with or without MALAT1 knockdown. (F,G) The capacity of spheroid formation was measured in ESCC cells with or without MALAT1 knockdown by detecting spheroid size (F) and number (G); scale bar, 100 μm. (H) ALDH1 activity was evaluated in the cells depicted in (C). The difference was assessed using one‐way ANOVA with the Tukey–Kramer *post hoc* test. Data are presented as the mean ± SD, *n* ≥ 3, **P < 0.01 vs. HECCs or Control.

### Knockdown of MALAT1 decreases the migration ability of ESCC cells

Cancer stem cells facilitate tumor metastasis, and the effects of MALAT1 on the cell migration of ESCC cells were further examined. As shown in Fig. 2A,B, knockdown of MALAT1 decreased the migration ability of ESCC cells. Therefore, these results demonstrate that lncRNA MALAT1 positively regulates the stemness of ESCC cells.

The article "Long noncoding RNA MALAT1 promotes the stemness of esophageal squamous cell carcinoma by enhancing YAP transcriptional activity" was retracted in 2023. Reasons: duplicated images; signs of a paper mill; unreliable results or conclusions.

**Figure 2:** Knockdown of MALAT1 decreases the migration ability of ESCC cells. (A, B) The migration ability of ESCC cells with or without MALAT1 knockdown was examined (A) and quantified (B); scale bar, 200 μm. The difference was assayed using one‐way ANOVA with the Tukey–Kramer *post hoc* test. Data are presented as the mean ± SD, *n* ≥ 3, **P < 0.01 vs. Control.

### Knockdown of MALAT1 enhances chemo‐ and radiosensitivity of ESCC cells

As CSCs are regarded as the root of tumor chemoresistance and radioresistance, the involvement of MALAT1 in chemo‐ and radiosensitivity of ESCC cells was further explored. As shown in Fig. 3A,B, knockdown of MALAT1 enhanced the chemosensitivity of ESCC cells. Additionally, the radiosensitivity of ESCC cells was promoted by knockdown of MALAT1 as well (Fig. 3C,D).

**Figure 3:** Knockdown of MALAT1 enhances chemo‐ and radiosensitivity of ESCC cells. (A, B) IC_50_ values were measured in ESCC cells with or without MALAT1 knockdown plus cisplatin treatment. (C, D) ESCC cells with or without MALAT1 knockdown were treated with 3.2 Gy·min^−1^ radiation followed by detecting the cell viability. The difference was assayed using one‐way ANOVA with the Tukey–Kramer *post hoc* test. Data are presented as the mean ± SD, *n* ≥ 3, *P < 0.05, **P < 0.01 vs. Control.

### MALAT1 directly binds to YAP, enhances YAP protein expression and increases YAP transcriptional activity

Following this, the mechanisms by which MALAT1 exerts its effects on the stemness of ESCC cells were explored. As the transcriptional factor YAP plays a critical role in the expansion of CSCs and lncRNA has been shown to regulate YAP activity 19, 20, 26, it is assumed that MALAT1 could regulate YAP transcriptional activity. As expected, knockdown of MALAT1 decreased YAP transcriptional activity, which is characterized by the decrease in 8xGTIIC‐luciferase plasmid activity (Fig. 4A). Consistently, knockdown of MALAT1 decreased expression of connective tissue growth factor, a target of YAP (Fig. 4B,C). Furthermore, knockdown of MALAT1 reduced YAP protein level (Fig. 4D). Additionally, RIP analysis showed that MALAT1 directly bound to YAP (Fig. 4E). Notably, the level of mRNA and promoter activity of YAP were unaffected by knockdown of MALAT1 (Fig. 4F,G). Overall, the obtained results indicate that MALAT1 directly binds to YAP protein, and not mRNA or promoter, and thus promotes YAP protein level and transcriptional activity.

The article "Long noncoding RNA MALAT1 promotes the stemness of esophageal squamous cell carcinoma by enhancing YAP transcriptional activity" was retracted in 2023. Reasons: duplicated images; signs of a paper mill; unreliable results or conclusions.

**Figure 4:** MALAT1 directly binds to YAP, enhances YAP expression and increases YAP transcriptional activity. (A) The luciferase activity of 8xGTIIC‐luciferase plasmid was determined in ESCC cells with or without MALAT1 knockdown. (B,C) The expression of connective tissue growth factor (CTGF), a target of YAP, was examined in the cells depicted in (A). (D) The protein level of YAP was detected in the cells described in (A). (E) The MALAT1 level pulled down by anti‐YAP was measured in ESCC cells. (F) YAP mRNA level was examined in the cells depicted in (A). (G) The promoter activity of YAP was determined in the cells described in (A). The difference was assayed using one‐way ANOVA with the Tukey–Kramer *post hoc* test. Data are presented as the mean ± SD, *n* ≥ 3, **P < 0.01 vs. Control or IgG.

### Overexpression of YAP rescues MALAT1 knockdown‐mediated inhibitory effects on ESCC cell stemness and migration

Finally, attempts were made to determine whether MALAT1‐mediated effects were indeed through YAP. Len‐YAP‐OE was infected in ESCC cells with Len‐MALAT1‐KD infection. The infection efficiency was validated via western blot analysis (Fig. 5A). As shown in Fig. 5B–D, overexpression of YAP saved the expression of stemness markers which was decreased by knockdown of MALAT1. Additionally, the reduced capacity of spheroid formation induced by knockdown of MALAT1 was partially nullified by YAP overexpression (Fig. 5E,F). From Fig. 5G, it can be noted that consistent results were observed in ALDH1 activity. Furthermore, MALAT1 knockdown‐mediated decrease of ESCC cell migration ability was attenuated by YAP overexpression (Fig. 6A,B). Moreover, the enhanced radiosensitivity induced by knockdown of MALAT1 was partially reversed by YAP overexpression (Fig. 6C,D). Hence, the current study demonstrates that the MALAT1–YAP axis positively regulates the stemness of ESCC cells.

**Figure 5:** Overexpression of YAP rescues MALAT1 knockdown‐mediated inhibitory effects on ESCC cell stemness. (A) The protein level of YAP was examined in ECSS cells with MALAT1 knockdown plus YAP overexpression or not. (B, C) The mRNA levels of stemness markers (SOX2 and Nanog) were measured in the cells depicted in (A). (D) The protein levels of stemness markers (SOX2 and Nanog) were detected in the cells described in (A). (E,F) The capacity of spheroid formation was measured in the cells depicted in (A) by detecting spheroid size (E) and number (F); scale bar, 100 μm. (G) ALDH1 activity was evaluated in the cells depicted in (A). The difference was assayed using one‐way ANOVA with the Tukey–Kramer *post hoc* test. Data are presented as the mean ± SD, *n* ≥ 3, *P < 0.05, **P < 0.01 vs. Control or IgG.

The article "Long noncoding RNA MALAT1 promotes the stemness of esophageal squamous cell carcinoma by enhancing YAP transcriptional activity" was retracted in 2023. Reasons: duplicated images; signs of a paper mill; unreliable results or conclusions.

**Figure 6:** Overexpression of YAP rescues MALAT1 knockdown‐mediated inhibitory effects on ESCC cell migration, chemo‐ and radiosensitivity. (A, B) The migration ability was examined (A) and quantified (B) in ESCC cells with MALAT1 knockdown plus YAP overexpression or not; scale bar, 200 μm. (C,D) Cell viability was detected in the cells depicted in (A) following by 3.2 Gy·min^−1^ radiation treatment. The difference was assayed using one‐way ANOVA with the Tukey–Kramer *post hoc* test. Data are presented as the mean ± SD, *n* ≥ 3, **P < 0.01 vs. Control or IgG.

## Discussion

In the current study, we identified the promoting roles of lncRNA MALAT1 in the stemness of ESCC cells by directly binding to YAP, enhancing YAP protein expression and increasing YAP transcriptional activity. Although the impellent roles of MALAT1 in regulating tumor stemness have been disclosed in colorectal cancer 27 and gastric cancer cells 28, to the best of our knowledge, we are the first to demonstrate the novel MALAT1–YAP axis in regulating the stemness of ESCC cells.

Long noncoding RNAs are first defined as ‘non‐functional genes’ that lack protein‐coding ability; nevertheless, increasing evidence reveals that lnRNAs hold an important biological role in tumorigenesis 29, 30. Although the oncogenic functions of lncRNA MALAT1 have been disclosed 10, 31, a few studies also showed tumor‐suppressive roles of MALAT1. For example, MALAT1 was identified as a target of phosphatase and tensin homologue (PTEN), which is responsible for the suppressive roles of PTEN in colon and breast cancers 32. Additionally, MALAT1 suppresses glioma progression via reduction of extracellular signal‐regulated kinase/mitogen‐activated protein kinase signaling activity and expression of matrix metalloproteinase 2 33. Furthermore, MALAT1 inhibits breast cancer metastasis via binding and inactivating the prometastatic transcriptional factor TEAD through a transgenic mouse model of breast cancer 11. These findings demonstrate that MALAT1 functions specifically in different types of cancers. In the current work, it has been found that MALAT1 exhibited a higher level in ESCC cells compared to HEECs and for the first time the oncogenic role MALAT1 in ESCC cell stemness was characterized.

Long noncoding RNAs fulfill their functions through specific interactions with other factors such as protein 23, mRNA 34 and DNA 26, and so a strategy to investigate the underlying mechanisms contributing to their functions is through exploring their partners. For example, the region of 1408–1867 nt of lncRNA uc.34 binds to the 592–759 aa region of CUL4A and inhibits CUL4A nuclear export, and this process hinders the CUL4A‐mediated ubiquitination of LATS1 in hepatocellular carcinoma 30. Spiniello *et al*. established a HyPR‐MS platform and efficiently elucidated the interactomes of lncRNAs MALAT1, NEAT1, and NORAD 35. Additionally, lncRNA THOR, a conserved cancer/testis lncRNA, interacts with IGF2BP1 and contributes to its mRNA stabilization activities 36. Here, we found that MALAT1 directly binds to oncogenic transcription factor YAP, increases YAP protein expression and enhances the stemness of ESCC cells. However, the mechanism by which MALAT1 regulates YAP protein expression is still unclear. It is speculated that MALAT1 might enhance YAP protein stability and suppress its degradation, but this needs further investigation. Also, further *in vivo* experiments should be carried out to prove this.

The article "Long noncoding RNA MALAT1 promotes the stemness of esophageal squamous cell carcinoma by enhancing YAP transcriptional activity" was retracted in 2023. Reasons: duplicated images; signs of a paper mill; unreliable results or conclusions.

Researchers have designed small molecules specifically targeting the MALAT1 ENE triplex and molecular probes for the treatment and investigation of MALAT1‐driven cancers 37, and constructed MALAT1‐specific antisense oligonucleotides and nucleus‐targeting TAT peptide cofunctionalized gold nanoparticles to inhibit cancer metastasis 38. The current study indicates the oncogenic role of the MALAT1–YAP axis in ESCC, implying that MALAT1 may be a novel target for ESCC treatment as well.

## Conflict of interest

The authors declare no conflict of interest.

## Author contributions

QY and JY conceived and designed the project, QY, TL JZ and YZ acquired the data, QY and JY analyzed and interpreted the data, and QY and JY wrote the paper.
